The article "The ubiquitin system: orchestrating cellular signals in non-small-cell lung cancer" was published in 2020. Journal: Cell Mol Biol Lett.

# The ubiquitin system: orchestrating cellular signals in non-small-cell lung cancer

**DOI:** 10.1186/s11658-019-0193-6

**Published:** 2020-01-16

**Authors:** Qiang Fan, Qian Wang, Renjie Cai, Haihua Yuan, Ming Xu

**Affiliations:** 1 Department of Oncology, Shanghai 9th People’s Hospital, Shanghai Jiao Tong University School of Medicine, 280 Mohe Road, Shanghai, China; 2 Department of General Surgery, Shanghai 9th People’s Hospital, Shanghai Jiao Tong University School of Medicine, 280 Mohe Road, Shanghai, China

**Keywords:** Ubiquitin, Ubiquitination, Deubiquitination, Cell signaling, Lung cancer

## Abstract

The ubiquitin system, known as a common feature in eukaryotes, participates in multiple cellular processes, such as signal transduction, cell-cycle progression, receptor trafficking and endocytosis, and even the immune response. In lung cancer, evidence has revealed that aberrant events in ubiquitin-mediated processes can cause a variety of pathological outcomes including tumorigenesis and metastasis. Likewise, ubiquitination on the core components contributing to the activity of cell signaling controls bio-signal turnover and cell final destination. Given this, inhibitors targeting the ubiquitin system have been developed for lung cancer therapies and have shown great prospects for clinical application. However, the exact biological effects and physiological role of the drugs used in lung cancer therapies are still not clearly elucidated, which might seriously impede the progress of treatment. In this work, we summarize current research advances in cell signal regulation processes mediated through the ubiquitin system during the development of lung cancer, with the hope of improving the therapeutic effects by means of aiming at efficient targets.

## Background

Lung cancer is one of the most common malignant tumors and the leading cause of cancer-related mortality in the worldwide [1]. Non-small-cell lung carcinoma (NSCLC) represents 85% of all lung cancers and patients’ 5-year survival rate is only about 18% [2, 3]. The major challenges in the treatment of lung cancer are metastasis and drug resistance [4, 5]. At present, there is still no effective solution for them because of our poor understanding of the molecular mechanisms of lung cancer. Increasing evidence indicates that proteasome inhibition has become an attractive and potential anticancer therapy due to the UPS, like other cellular pathways, being critical for the proliferation and survival of cancer cells [6, 7]. For developing novel therapeutic approaches to treat lung cancer, it is important to deeply comprehend the different cell signaling and intricate mechanisms orchestrated via the ubiquitin pathway in association with lung cancer [4].

The article "The ubiquitin system: orchestrating cellular signals in non-small-cell lung cancer" was published in 2020. Journal: Cell Mol Biol Lett.

The UPS, which consists of a 26S proteasome and a small ubiquitin molecule, is a major protein degradation system which regulates a number of cellular functions, and is implicated in most of the cell signaling activities [8–10]. In recent years, dysregulation of various UPS components has been observed in cancer diseases including lung cancer [11–14]. Ubiquitination (and its reversal, deubiquitination) is one of the PTMs and plays important roles in regulation of a large number of cellular processes [15, 16], including cell cycle regulation [17, 18], apoptosis [19, 20], DNA damage [21–23] and immune functions [20, 24, 25]. Likewise, dysregulation of ubiquitination also results in aberrant activation or deactivation of signaling pathways. Thus, better understanding of the regulation mechanisms may ultimately lead to novel therapeutic modalities in lung cancer by targeting the ubiquitin pathway.

Here, we provide a comprehensive overview about ubiquitination and deubiquitination of the main components in cell signaling (i.e., PI3K-AKT-mTOR and RAS-RAF-MEK-ERK), which have been found to be regulated primarily in lung cancer. We also highlight the recent progress in our understanding of the molecular mechanisms by which cancer-associated proteins mediate cell signaling networks through the ubiquitin system.

### Ubiquitin, ubiquitination and deubiquitination

Ubiquitin is found in all known eukaryotic organisms and it has a highly conserved 76 amino acid sequence that undergoes covalent attachment to lysine residues in target proteins via isopeptide linkage [15]. A single ubiquitin molecule contains 7 lysine residues (K6, K11, K27, K29, K33, K48, and K63) to which another ubiquitin can be ligated, resulting in different types of poly-ubiquitin chains involved in diverse cell processes [26, 27]. However, the poly-ubiquitin chain in which each additional ubiquitin molecule is linked to lysine 48 (K48) of the previous ubiquitin plays a main role in proteasome degradation [27], whereas K63-linked ubiquitin chains have been thought to participate in regulating various proteasome-independent cellular functions, including NF-κB signaling, DNA damage repair, ribosomal function, and intracellular trafficking [28, 29].

The process of ubiquitination requires the help of at least three different enzymes: ubiquitin-activating enzyme E1, ubiquitin-conjugating enzyme E2 and ubiquitin ligase E3 [30–32]. E3 ubiquitin ligases are critical in the UPS, as they mediate the specificity of substrate recognition and allow the transfer of activated ubiquitin from E2 enzymes to the target protein [33, 34]. Structurally, E3s can be divided into HECT-type E3s with a HECT domain which forms a thiolester bond with ubiquitin and then conjugates it to the substrate [35, 36], RING finger-containing E3s containing RING and U-box domains [37–39], RING-between-RING family members which have a RING1-in-between RING-RING2 motif [40]. Moreover, deubiquitination, known as a reverse process of ubiquitination, is also a complex enzymatic system responsible for removing ubiquitin from a substrate [41]. The isopeptide bond between ubiquitin and its substrate can be cleaved by the specific DUBs to produce monoubiquitin for recycling [16, 42–44]. Recently, more than 100 DUBs have been found that can be divided into five subfamilies: USP, OTU, MJD, UCH and JAMM/MPN metalloproteases [16, 44].

The article "The ubiquitin system: orchestrating cellular signals in non-small-cell lung cancer" was published in 2020. Journal: Cell Mol Biol Lett.

To date, increasing evidence has shown that ubiquitin E3 ligase and deubiquitination enzymes are directly involved in the regulation of tumor formation and metastasis of lung cancer, especially through the RAS-RAF-MEK-ERK and PI3K-AKT-mTOR signaling pathways, in which the ubiquitination of key signal nodes determines the biological and biochemical processes of tumor cells (Table 1). Below, we summarize the molecular mechanism mediated through the ubiquitin system in the development of lung cancer, and hope to supply more cues for the therapeutic strategy.

**Table 1:** A list of ubiquitin E3 ligases and deubiquitination enzymes that have been found in regulation of associated genes in NSCLC

Genes	E3 Ligases	DUBs	Main function in lung cancer through the ubiquitin system	Ref
EGFR	c-Cbl, Cbl-b	USP8, USP2a, AMSH	EGFR is often overexpressed and mutated in lung cancer, especially in non-small cell lung cancer. Mono-ubiquitinated or poly-ubiquitinated EGFR upon EGF stimulation do not affect tyrosine kinase activity or signaling capacity but play a critical role in lysosomal targeting. Ubiquitination of EGFR can facilitate its endocytosis and degradation. Disruption of the negative regulatory system is associated with lung carcinogenesis, while deubiquitinating enzymes can reverse this modification and hence oppose endosomal sorting and lysosomal degradation in non-small cell lung cancers.	[45–48]
Ras	NEDD4–1, Rabex5, βTrCP1	–	RAS proteins are central mediators downstream of growth factor receptor signaling and therefore are critical for cell proliferation, survival, and differentiation. KRAS and NRAS mutations are more commonly found in lung cancers with adenocarcinoma histology. However, the ubiquitin system controls the subcellular localization and stability of Ras family protein in cancer cells, thereby contributing to the occurrences of tumor formation or metastasis.	[49–51]
Raf	RNF149, CHIP, TRAF2	–	Function as protein kinase to phosphorylate MAP 2 K1 directly, and thereby contributes to the MAPK signal transduction. Somatic mutations in BRAF, especially at valine 600 (V600), commonly occurred in non-small cell lung cancer, and this mutated BRAF can escape from degradation via the ubiquitin proteasome system. However, K63-linkaged poly-ubiquitination of BRAF impairs the activity in BRAF-mediated ERK activation, which induced by RNF149 E3 ligase. TRAF2 is a novel E3 ligase of BRAF K48-linkaged poly-ubiquitination which affects its stability.	[52–54]
PTEN	NEDD4–1, WWP2, XIAP, CHIP	USP7, USP13	It functions as a tumor suppressor that is mutated in a large number of cancers at high frequency and subcellular localization has been strongly implicated in the regulation of the PI3K/AKT pathway. Loss of PTEN expression is common in lung adenocarcinoma. Mono-ubiquitination and poly-ubiquitination of PTEN can be induced by NEDD4–1, WWP2, XIAP or CHIP, and deubiquitinated by USP7 or USP13 leading to its nuclear exclusion. Mono-ubiquitination of one of either Lys-13 or Lys-289 amino acid is sufficient to modulate PTEN compartmentalization. Phosphorylation of PTEN at Tyr-336 protects it from ubiquitin-mediated degradation probably by inhibiting its binding to NEDD4–1.	[55–58]
AKT	CHIP, BRCA1, NEDD4–1, Skp2, TRAF6, TRAF4	CYLD	The AKT kinase, which regulates many cell processes, plays a critical role in the development of multiple cancer types and tumorigenesis. In lung cancer, it is abnormally activated via the post-translational modification, including phosphorylation, ubiquitination and sumoylation, thereby impairing its subcellular location and cell signaling transduction. The ubiquitin system induces the ubiquitination of AKT with different lysine-linkage types either for the proteasome degradation or for the function alteration to affect the cell signaling transduction and control the evolution of cancer cells.	[59–61]
mTOR	Fbxw7, TRAF6	–	It functions as the main component of mTORC1 and mTORC2, and mTORC1 exerts a feedback control on upstream growth factor signaling including PI3K/AKT and MAPK signaling. Upon the stimuli of amino acid, the K63-likaged poly-ubiquitination of mTOR indirectly induced by TRAF6 promotes the mTORC1 activation to accelerate downstream signaling in non-small cell lung cancer. However, the K48-linkaged poly-ubiquitination of mTOR impacts both of mTORC1 and mTORC2 activities due to the proteasome degradation induced by Fbxw7.	[62–65]

The article "The ubiquitin system: orchestrating cellular signals in non-small-cell lung cancer" was published in 2020. Journal: Cell Mol Biol Lett.

### Ubiquitination in RAS-RAF-MEK-ERK pathway

The RAS-RAF-MEK-ERK pathway, mainly composed of Raf kinase, Ras-GTPase, MEK, and ERK, is the most characteristic pathway in cell biology involved in regulating cell proliferation, differentiation and apoptosis [66]. This signaling pathway is usually activated by a variety of growth factors, chemokines, polypeptide hormones, neurotransmitters, and phorbol esters through their cognate RTKs [67] and GPCRs [66], or by direct activation of PKC [68, 69]. Dysregulation of the ERK pathway, mainly caused by constitutive activation of Ras and Raf, has been well established in human malignancies [70] **(**Fig. 1**)**. The activation of ERK1/2 promotes cell survival and chemotherapeutic resistance in lung cancer and greatly contributes to the development of NSCLC [71]. Likewise, ERK-dependent serine/threonine phosphorylation of specific substrates is essential for the ubiquitination and degradation process [72].

**Fig. 1:** Ubiquitination on RAS-RAF-MEK signal. Upon EGF or other growth factors stimulation, activated Ras-GTP enhances the transcripts of NEDD4–1 which promotes the ubiquitination on all three forms of Ras-GTP and PTEN for the proteasome degradation to accelerate the downstream signaling activation. Rabex, to some extent as a ‘break’, can ligate mono- or poly-ubiquitin (K63-link) to HRas or NRas, but not KRas, which promotes their endosome localization and lysosome degradation, thereby limiting the transformation of Ras-GTP from Ras-GDP to suppress the phosphorylation activation of ERK. Likewise, BRAF and CRAF can be ubiquitinated by RNF149 and CHIP, respectively, and be degraded by the proteasome to decelerate MEK/ERK activation, which attenuates the increase in cell growth. Following EGF stimulation, RING domain E3 ubiquitin ligases c-Cbl or Cbl-b, with the assistance of Grb2, induces mono- or poly-ubiquitination (K63-link) of EGFR and mediates the endosomal sorting and trafficking events, in which process the mono-ubiquitinated EGFR is trapped within ILVs of multivesicular bodies (MVBs), whereas poly-ubiquitinated forms remaining in the MVBs are deubiquitinated by DUB enzymes USP8, USP2a or AMSH to escape the ILVs trapping and lysosome degradation. Instead, the non-ubiquitinated EGFR forms are recycled to the cell membrane for the downstream signal activation

### Ubiquitination controls Ras protein level and subcellular localization

Ras is a small GTPase that is activated by various cell-surface molecules, and membrane localization is essential for its activation [73]. All three Ras isoforms, H-Ras, K-Ras (two splice variants, K-Ras4A and K-Ras4B), and N-Ras reside in the plasma membrane and switch on/off for the downstream signal transduction [74], whereas the ubiquitination of Ras has been shown to control Ras protein turnover as well as its subcellular localization [50]. Rabex-5 (also known as RabGEF1) functions as an E3 ligase for mediating Ras (H-Ras and N-Ras, but not K-Ras) ubiquitination to promote Ras endosomal localization, and further leads to the suppression of ERK activation [75]. Meanwhile NEDD4–1 can regulate Ras-GDP level of all three forms and subsequently drives PTEN degradation, leading to tumor processes [76] **(**Fig. 1**)**. Smurf2 and UbcH5 as a critical E3 and E2, respectively, are important in maintaining K-Ras protein stability, and targeting such a complex was supposed to be a unique strategy to degrade mutant K-Ras^G12/V or C^ to kill cancer cells [51]. However, knock-down Smurf2 can accumulate the F-box protein βTrCP1 which mediates poly-ubiquitination and proteasome-dependent degradation of Ras [51, 77]. H- and N-Ras, but not K-Ras, are subjected to mono- and K63-linked di-ubiquitination, and stabilize their associations with the endosome, resulting in a change in the signaling output [49], while K-Ras shows only minor or transient association with the endosome [78]. However, K147 in K-Ras or H-Ras was identified as one of the major ubiquitination sites; the modification of it increases the fraction of GTP-bound Ras and more efficiently activates Raf and PI3K to enhance its tumorigenic activity [50]. Intriguingly, monoubiquitination on K147 in K-Ras does not affect protein localization, but rather impedes GAP-mediated GTP hydrolysis and promotes the association with downstream effectors [79, 80]. In lung cancer disease, the sustained activation of ERK is a common event and frequently contributes the tumor growth and even the metastatic processes; therefore it might be an efficient way to abolish the enhanced Ras protein level or Ras-GTP activity by inhibiting its E3 ubiquitin ligase (i.e. NEDD4–1) to suppress the tumor progress.

The article "The ubiquitin system: orchestrating cellular signals in non-small-cell lung cancer" was published in 2020. Journal: Cell Mol Biol Lett.

The direct deubiquitination process of Ras has not been described in any cancer or other diseases. As reported, carboxyl-terminal CAAX motifs in Ras are essential for its activity and proper membrane localization, and can be cleaved by RCE1 [81], whereas RCE1 can be down-regulated by the deubiquitinating enzyme USP17, a process that occurs in the ER, through removing the functional K63 polyubiquitin chains of RCE1 [81, 82]. As a consequence, it blocks Ras membrane localization and activation, thereby inhibiting phosphorylation of the downstream kinases MEK and ERK [81]. Intriguingly, USP17 impedes EGF-induced H-Ras and N-Ras but not K-Ras membrane trafficking, no matter whether wild-type Ras or oncogenic mutants [81–83]. Suppression of USP17 inhibits the abilities of tumorigenesis and invasion of NSCLC cells in vitro and in vivo [84]. In clinical practice, USP17 was always observed over-expressed in both squamous and adenocarcinoma NSCLC tissues. Patients with USP17-positive tumors had significantly reduced recurrence-free survival and USP17 mRNA level positively correlated with NSCLC distant metastasis [85]. USP17 depletion can not only block the proliferation of NSCLC cells with EGFR wild-type, but also those bearing active mutations of EGFR or TKI resistant mutations [86]. This evidence suggests that USP17 may ultimately enhance the Ras activity to promote the tumor processes in NSCLC and could be a great potential therapy target for drug development for the treatment of NSCLC.

### Different Raf proteins play a distinct role in the cell signaling pathway

As the receptor tyrosine kinase effecter in the ERK pathway, Raf consisting of ARAF, BRAF, and CRAF shows a serine/threonine kinase activity, relevant to tumorigenesis, including cell proliferation, survival, invasion, and angiogenesis [54]. The three Raf proteins have a similar structure and all are considered to be oncogenic, but they execute distinct properties for MEK phosphorylation and activation [74]. Intriguingly, complex formation by these different isoforms play a critical role in their activation, particularly in response to RAF inhibitors, and BRAF/CRAF complexes seem to be stabilized by ARAF in cells, thereby regulating cell signaling to ensure signaling efficiency [87].

BRAF is modified by K63-linked polyubiquitination at K578 through gain of a constitutively active mutation (V600E, which renders the constitutive activation of BRAF and is responsible for more than 90% of somatic mutations in human tumors) under EGF stimulation [52]. Substitution of BRAF lysine 578 with arginine (K578R) weakened K63 polyubiquitination and inhibited BRAF-mediated ERK activation [88]. However, the specific E3 ligase(s) and deubiquitinating enzyme(s) controlling the positive and negative regulation of BRAF K63-linked polyubiquitination still need to be further identified [52]. RNF149, as a RING domain-containing E3 ubiquitin ligase, is involved in control of gene transcription, translation, cell adhesion, cytoskeletal organization or epithelial development. It is an authentic E3 ligase of wild-type BRAF, but not of mutant BRAF (V600E), and induces BRAF degradation through the ubiquitin proteasome system and thereby reduction of MEK/ERK activity [53] **(**Fig. 1**)**. TRAF2 is a novel E3 ligase of BRAF K48-linked ubiquitination. TRAF1 binding with TRAF2 could decrease BRAF K48-linked ubiquitination but not affect K63-linked ubiquitination. TRAF1 seems to serve as a ‘break’ for TRAF2 driving BRAF degradation, which activates MEK and ERK mediation of lung cancer cell growth, apoptosis or lung tumorigenesis [89] (Fig. 1). Therefore, blocking TRAF1 using appropriate chemical drugs to release TRAF2 might also be an ideal way to inhibit the sustained MEK/ERK activation in NSCLC.

The article "The ubiquitin system: orchestrating cellular signals in non-small-cell lung cancer" was published in 2020. Journal: Cell Mol Biol Lett.

CRAF (also termed Raf-1), normally residing in the cytoplasm as an inactive kinase, is activated by GTP-Ras and recruited to the cell membrane [90, 91]. This activation process is tightly regulated by various factors including kinases (e.g. ERK, Src, AKT, PKC), phosphatases (e.g. PP2A, PP1, PP5) and proteins that directly bind to CRAF (e.g. 14–3-3, RKIP, Hsp90, KSR) [90, 92]. Nevertheless, autophosphorylation of serine 621 (S621) is essential to ensure the correct folding and stability of the CRAF protein, which prevents it from being degraded by CHIP (carboxy terminus of Hsc70 interacting protein) [91]. Although CHIP is an identified E3 ubiquitin ligase of CRAF, it is not unique to induce the degradation of S621 non-phosphorylated CRAF [91].

### Ubiquitination of EGFR is involved in endosomal sorting and lysosome degradation

EGFR (also termed as HER1), one of RTKs of the ErbB family, is a transmembrane glycoprotein with cytoplasmic kinase activity that regulates signaling pathways to control cellular proliferation [93]. Mutation of EGFR has been strongly implicated in the pathogenesis of many human malignancies, especially in NSCLC [45, 94, 95]. The basic signal mechanism is that growth factors (e.g. EGF, FGF, PDGF and TGF-α) trigger membrane EGFR homo- and/or heterodimerization and autophosphorylation on key cytoplasmic residues, leading to receptor hyperactivity [93, 96]. Further, the phosphorylated EGFR recruits adapter proteins such as GRB2, which in turn activates complex downstream signaling cascades [97, 98], including the RAS-RAF-MEK-ERK, PI3K-AKT-mTOR, and probably the NF-κB signaling cascade [96, 98].

As reported, most cell surface receptors, including RTKs such as EGFR and β2AR, can be internalized and undergo rapid clathrin-dependent or -independent endocytosis which is required for maintenance of regulated receptor trafficking and kinase signaling [99, 100]. More compelling evidence has proved that ubiquitination is a major posttranslational modification of EGFR that controls the endosomal sorting and trafficking of diverse signaling receptors after endocytosis [46, 99]. In that process, endosomal protein ESCRT complexes I, II, and III, each containing a ubiquitin binding domain, and Hrs, which might deliver ubiquitinated cargo to the outer membrane of the late endosome, are thought to participate in trapping EGFR within ILVs of multivesicular bodies (MVBs) that are destined for subsequent degradation in the lysosome, thereby preventing their recycling to the plasma membrane [47, 48] (Fig. 1).

The article "The ubiquitin system: orchestrating cellular signals in non-small-cell lung cancer" was published in 2020. Journal: Cell Mol Biol Lett.

RING domain E3 ubiquitin ligases c-Cbl and Cbl-b, with the assistance of Grb2, induce ubiquitination of EGFR following EGF stimulation, which has been implicated in regulation of both its localization and stability [48, 101]. Multiple monoubiquitination of activated EGFR is thought to be involved in endocytic trafficking, and even a single ubiquitin is sufficient for both receptor internalization and degradation [47]. However, quantitative mass spectrometry demonstrated that multiple lysines in the kinase domain of EGFR could be primarily conjugated to K63-linked polyubiquitin chains for the endosomal sorting process and lysosome degradation [48]. Nevertheless, the further experiments implied that EGFR ubiquitination is not necessary for clathrin-mediated internalization, which might be controlled by multiple kinase- and ubiquitination-dependent and -independent mechanisms [102]. Conversely, endosomal DUBs such as USP2a, USP8/UBPy and AMSH reverse this modification and hence oppose endosomal sorting and lysosomal degradation [103–105]. Controversially, UBPy and AMSH may either accelerate or inhibit degradation of EGFR upon EGF stimulation, which due to the distinct catalytic or regulatory domain in their structures differentially control the EGFR turnover [45, 106, 107]. Moreover, USP2a, which localizes to early endosomes, is over-expressed in NSCLC and shows an oncogenic property through increasing the plasma membrane-localized EGFR, as well as decreasing the internalized and ubiquitinated EGFR [104] **(**Fig. 1**)**.

In addition, the functional defects of EGFR with specific mutations (L858R, del746–750 or L858R + T790 M) in NSCLC cells can be impaired, probably due to a propensity of the mutants to heterodimerize with HER2, thereby evading c-Cbl-mediated ubiquitination and subsequent sorting to degradation in lysosomes [108]. Intriguingly, the E3 ligase CHIP could selectively interact with and degrade the EGFR mutants such as G719S, L747_E749del A750P or L858R and inhibited tumor cell proliferation and xenograft growth of EGFR mutant but not EGFR WT cell lines, which might provide novel therapeutic strategies for overcoming the EGFR-TKI resistance in lung adenocarcinoma [109]. Taken together, this evidence suggested that it could be an efficient manner to promote WT- or Mut- EGFR internalization and ubiquitination to impede its membrane localization via targeting USP2a, which could attenuate the activation of ERK signaling and thereby suppress the cancer processes in NSCLC.

### Ubiquitination in PI3K-AKT-mTOR pathway

The PI3K-AKT-mTOR signal is an intracellular signaling pathway and has a critical role in the regulation of the ubiquitin-proteasomal system and autophagy in mammalian cells [110, 111]. PI3K-AKT-mTOR pathway activation can be mediated by specific aberrations in PIK3CA, PIK3R1, AKT, LKB1, TSC1/2, EGFR or PTEN [112]. Many known factors can also enhance the PI3K-AKT-mTOR pathway including EGF [113], shh [114, 115], insulin [116], and IGF-1 [114]. Under the condition of stimuli, PI3K phosphorylates PIP2 to create PIP3 and recruits AKT to the plasma membrane to active PDK1 and mTOR complex which phosphorylates 4E-BP1 and p70 ribosomal S6 kinase that trigger ribosome biogenesis and translation in cell growth and division [61, 117] **(**Figs. 2&3).

The article "The ubiquitin system: orchestrating cellular signals in non-small-cell lung cancer" was published in 2020. Journal: Cell Mol Biol Lett.

**Fig. 2:** Ubiquitination on PI3K-AKT signal**.** Under the conditions of growth factor stimuli, such as insulin, activated RTKs recruit IRS1 (insulin receptor substrate 1) for binding and activation of p85-p110 heterodimers (PI3K). With the assistance of phosphatase PTPL1, free p85β is ubiquitinated by Fbxl2 and degraded through the proteasome system to block its competition with p85-p110 heterodimers binding to IRS1, thereby promoting activation of the PI3K-AKT signal. The p110 subunit of PI3K catalyzes the conversion of PIP2 to PIP3, which recruits AKT to the plasma membrane for activation through PDK1 and PDK2. In that process, activation of AKT is inhibited by PTEN through conversion of PIP3 to PIP2 to restraint the downstream events, i.e., K48-linked polyubiquitination on phosphorylated AKT is triggered by E3 ligases CHIP, BRCA1, MULAN or TTC3 for proteasome degradation, but K63-linked AKT is induced by NEDD4–1, Skp2 and TRAF6 to mediate its nuclear localization for further activation of the PI3K-AKT signal. However, TRAF4 is the main effector for AKT K63-linked ubiquitination and promotes EGF-induced AKT membrane recruitment in human lung cancer cells to induce tumorigenic properties. Deubiquitinating enzyme CYLD plays a tumor suppressor role in inhibiting AKT activity by removing AKT K63-linked ubiquitin chains and serves as a negative regulator for AKT-mediated tumorigenesis. Ubiquitinated PTEN with poly-ub chains is usually degraded by the proteasome system, while partial mono-ubiquitinated forms translocate into the nucleus to escape proteasome degradation, mediated by NEDD4–1, WWP2, XIAP and CHIP E3 ligase. However, this progress can be reversed by deubiquitinating enzymes USP7 and USP13 to deactivate the PI3K-AKT signal

**Fig. 3:** Ubiquitination on mTOR signal affects the cross-talk between RAS-RAF-MEK and PI3K-AKT-mTOR pathways**.** TSC2 and mTORC1 as the downstream sensor receive many inputs from both RAS-RAF-ERK and PI3K-AKT signaling to activate S6K and 4E-BP1 for mRNA translation and protein synthesis, as well for inhibition of autophagy. Meanwhile, activated mTORC1 can enhance the RAF-ERK signaling through feedback inhibition of PI3K but not of AKT or mTORC2. In this pathway, Fbxw7 is responsible for recognizing mTOR and executing the ubiquitination (K48-Ub chains) for further proteasome degradation to reduce the activity of mTORC1 and mTORC2. Upon the stimulation of amino acid, K63-linked ubiquitin chains on mTOR are essential for activation of mTORC1, which is triggered by TRAF6 with the assistance of p62 and adaptor protein Raptor. However, Raptor, an essential component of mTORC1, can be poly-ubiquitinated and deubiquitinated by the DDB1-Cul4 complex and UCH-L1, respectively, thereby impairing the activity of mTORC1 and downstream signaling

The article "The ubiquitin system: orchestrating cellular signals in non-small-cell lung cancer" was published in 2020. Journal: Cell Mol Biol Lett.

### Ubiquitination on the p85 subunit contributes to the PI3K signaling cascade

In lung cancer, the PI3K pathway is frequently dysregulated due to genetic alterations [118]. PI3K is a family of lipid enzymes that specifically phosphorylate the 3′-hydroxyl group of phosphatidylinositols and phosphoinositides on membranes [119]. Classical PI3K is composed of a p85 (p85α, p85β and p55γ) regulatory subunit and a p110 catalytic subunit [120, 121]. A certain amount of p85, which lacks intrinsic kinase activity, is necessary for PI3K to bind phospho-tyrosine docking sites at the cell membrane [122], while excessive free p85 could compete with p85-p110 heterodimers binding to IRS1, a process which inhibits the PI3K activity and its downstream signaling. Fbxl2, a member of the F-box protein family which usually forms the ubiquitin E3 complex with Skp1, Rbx1 and Cul1, specifically binds p85α and p85β, but not p110 [122]. However, Fbxl2 can only induce the degradation of tyrosine-dephosphorylated p85β triggered by the phosphatase PTPL1, which inhibits the excessive free p85 contacting IRS1, leading to an increase in the binding of p85-p110 heterodimers to IRS1 and enhancement of the PI3K signaling cascade [122] (Fig. 2). Therefore, suppressing Fbxl2 activity to maintain free p85 forms in cells will help to inhibit the aberrant activation of PI3K/AKT signaling to some extent in NSCLC.

### Different ubiquitin linkages of AKT mediate a diverse cell signaling pathway

AKT, also known as PKB, is a serine/threonine protein kinase involved in various signaling transduction pathways [123]. AKT, as one of the major downstream effectors of PI3K, plays a vital role in the promotion of cell proliferation and preventing the cell from entering the apoptotic pathway by interacting with caspase-9 and Bcl2 [124]. The inactivation of PTEN and RAS also can stimulate AKT activation, and excessive activation of AKT was suggested to be a poor prognostic factor for early stage NSCLC patients [61]. However, ubiquitination is completely essential for AKT signaling activation. For instance, K63-linked ubiquitination mediated by NEDD4–1 [125], Skp2 [59] and TRAF6 [59, 126], which itself could be negatively mediated by c-Cbl [127], induces AKT activation via promoting plasma membrane translocation and nuclear translocation. Converse evidence suggests that TRAF4, but not Skp2, is required for AKT K63 ubiquitination and promotes EGF-induced AKT membrane recruitment in human lung cancer cells to induce tumorigenic properties [60], but TRAF6 is unnecessary for EGF-induced AKT activation [59, 60]. In contrast, K48-linked ubiquitination mediated by CHIP, BRCA1, MULAN and TTC3 triggers the proteasomal degradation of phosphorylated AKT to terminate its activation **[**29, 111, 128–130**]**. Nevertheless, the ubiquitination of AKT can be reversed by CYLD, which is a deubiquitinating enzyme and plays a tumor suppressor role in inhibiting AKT activity by removing AKT K63-linked ubiquitin chains and serves as a negative regulator for AKT-mediated tumorigenesis or lung fibrosis [131] **(**Fig. 2**)**. It is worth mentioning that deubiquitinase CYLD and E3 ubiquitin ligase Itch are able to form a complex by interaction through “WW-PPXY” motifs, and sequentially cleave K63-linked ubiquitin chains for catalyzing K48-linked ubiquitination on Tak1 to terminate inflammatory signaling via TNFs [132]. Deficiency in either Itch or CYLD will lead to the chronic production of cytokines specifically generated by tumor-associated macrophages, which further contributes to the aggressive growth of lung carcinoma [132]. Additionally, CYLD overexpression can block TRAIL-induced NF-κB activation directly, and consequently increase TRAIL-induced apoptosis in lung cancer cells [133]. This evidence revealed that TRAF4, SKP2, NEDD4–1 or TRAF6, but not CYLD, could be an ideal target for drug development and NSCLC therapy.

The article "The ubiquitin system: orchestrating cellular signals in non-small-cell lung cancer" was published in 2020. Journal: Cell Mol Biol Lett.

### PTEN has always been targeted by the ubiquitin system

PTEN, as a famous tumor suppressor, directly dephosphorylates phosphoinositides to antagonize the PI3K-AKT/PKB signaling pathway and thereby modulates protein synthesis, cell cycle and cell survival [134, 135]. PTEN attenuates PI3K signaling by directly binding pleckstrin homology domains of specific signaling proteins to dephosphorylate PIP3 to PIP2 [136, 137]. Loss of PTEN increases the phosphorylation of AKT and deregulates PI3K signaling, which in turn enhances cell survival [138–141]. However, PTEN is not frequently targeted at the genetic level in the development of lung cancer, and mutations of the PTEN gene in patients harboring NSCLC have been reported in 8 to 17% [135]. On the other hand, PTMs of PTEN that regulate its enzymatic activity, interaction with other proteins and subcellular localization have been strongly implicated in the regulation of the PI3K/AKT pathway [57, 135, 142, 143]. The PTEN protein level is controlled to a large extent by E3 ligase-mediated UPS degradation [55]; therefore, stabilizing PTEN protein level is a promising therapeutic strategy for most cancer diseases including NSCLC. NEDD4–1 [58, 144], WWP2 [145], XIAP [146] and CHIP [55] have been reported to be responsible for PTEN turnover (Fig. 2). Among them, NEDD4–1 was first identified as an E3 ubiquitin ligase that regulates stability of PTEN [144] (Fig. 1 and Fig. 2), and plays a critical role during the development of NSCLC [135]. NEDD4–1 is over-expressed in 80% of NSCLC tumors and correlates with the deficiency of PTEN protein [56, 135, 147]. In the mechanism, NEDD4–1 physically interacts with PTEN and leads to both mono- and poly-ubiquitination of PTEN at K289 and K13 sites [57]. However, mono-ubiquitination of PTEN appears to be a limited step for proteasome degradation while it is crucial for its nuclear import [57] (Fig. 2).

USP7 (also known as HAUSP) and USP13, as specific DUBs of PTEN, reversely regulate the stability of PTEN. USP7 was first found to be able to stabilize p53 through its intrinsic deubiquitinating enzyme activity in the lung cancer cell line H1299 [148]. In acute promyelocytic leukemia, the removal of either K289 or K13 mono-ubiquitin from PTEN by USP7 restrains PTEN nuclear localization without affecting its protein level [149]. Despite that, PML opposes the activity of USP7 towards PTEN through a mechanism involving the adaptor protein DAXX (death domain-associated protein) [149]. USP13 functions as a tumor suppressor mainly through reversing PTEN poly-ubiquitination and stabilizing PTEN protein levels via its deubiquitination action [150]. However, the functions of USP13 in lung cancer have not yet been elucidated. More interestingly, ataxin-3, as one member of the Josephin family DUBs, can enhance the transcription level of PTEN probably through stabilizing its specific transcriptional activators to down-regulate AKT phosphorylation and PI3K signaling in NSCLC [143].

### Cross-talk between PI3K-AKT-mTOR and RAS-RAF-MEK signal

The RAS-MEK-ERK and PI3K-AKT-mTOR pathways can negatively or positively regulate each other’s activities, in which the mammalian target of rapamycin (mTOR) is a core component sensor. mTOR, a serine/threonine protein kinase and the catalytic subunit of complexes including mTORC1 and mTORC2, has been identified as the downstream target of the PI3K/AKT pathway that regulates processes including mRNA translation, proliferation, and survival [151, 152]. The activity of mTORC1 can be regulated through the function of tuberous sclerosis complex (TSC1 and TSC2) activated by membrane localized AKT and enhances the GTPase activity of the mTOR activator Rheb [62, 153], thereby promoting cell growth via up-regulation of protein synthesis through activation of 4E-BP1 and p70S6 kinase [63, 154] (Fig. 3). However, inhibition of mTORC1 can lead to RAS-MEK-ERK activation through PI3K-dependent feedback but not mTORC2, AKT or targets of downstream of AKT in human cancer [62], which reveals an alternative signal whereby phosphorylation at Ser259 of Raf by AKT deactivated and inhibited the signal cascade of RAS-MEK-ERK [155] (Fig. 3). Evidence has shown that inhibition of the mTOR pathway represents a promising therapeutic approach for lung cancer [64, 156, 157].

The article "The ubiquitin system: orchestrating cellular signals in non-small-cell lung cancer" was published in 2020. Journal: Cell Mol Biol Lett.

Like AKT, ubiquitination also plays a key role in regulation of the mTOR pathway. E3 ubiquitin ligase TRAF6 is necessary for mTORC1 translocation to the lysosomes, and the TRAF6-catalyzed K63 ubiquitination of mTOR regulates mTORC1 activation through p62 upon amino acid stimulation [63]. Nonetheless, mTOR can be degraded by the ubiquitin proteasome pathway and Fbxw7 is an mTOR regulator that altered its expression in a manner opposite to mTOR, which affects the activity of both mTORC1 and mTORC2 [65, 158]. Moreover, Rictor as an essential component of mTORC2 could also be directly mediated by Fbxw7 for ubiquitination and proteasome degradation, which thereby impairs the AKT activation and downstream signaling [159]. Under mitochondrial stress, maintenance of mTORC1 activity requires the ubiquitination of mTOR at K2066 and K2306 catalyzed by Parkin, which in turn promotes cell survival and growth [160]. In addition, UCH-L1 as a ubiquitin hydrolase of Raptor has a critical role in regulation of the dichotomy between mTORC1 and mTORC2 signaling, and it impairs mTORC1 activity toward S6 kinase and 4E-BP1 while increasing mTORC2 activity toward AKT [161] (Fig. 3).

## Therapies and prospects

Cell signaling responses play an important role in regulating cell characteristics. However, the key regulation nodes function as a signaling ‘switch’ to mediate cell processes. Meanwhile, the ubiquitination system intricately regulates activation and inactivation of these signaling pathways. The examples described here illustrate that the PI3K-AKT-mTOR and RAS-RAF-MEK pathways are subjected to the ubiquitin regulation in lung cancer, and the ubiquitination on those signaling nodes directly orchestrates the cell signal transduction positively or negatively. Although some of the E3s or DUBs mentioned above have shown some potential as drug targets for the treatment of NSCLC, more experimental evidence and clinical trials are needed to identify the effects.

The article "The ubiquitin system: orchestrating cellular signals in non-small-cell lung cancer" was published in 2020. Journal: Cell Mol Biol Lett.

Given this, inhibition of the ubiquitin system, including proteasome, E1, E2, E3 and DUB, has been developed and proven a very effective treatment in multiple malignancies in addition to NSCLC. For example, bortezomib (PS-341), the first proteasome inhibitor approved by the FDA for the treatment of multiple myeloma, has been tested in numerous NSCLC models in vitro and in vivo, and shows an active effect against NSCLC cells. In preclinical studies, bortezomib inhibits the proteasome activity and further affects the function of numerous proteins involved in processes such as cell-cycle control, apoptosis, angiogenesis, and chemoresistance [162–165]. Currently, phases I and II studies show promising results in combination therapy for NSCLC through combining bortezomib with available chemotherapeutic agents or targeted therapy [166–168], such as carboplatin/bevacizumab [166], paclitaxel/carboplaitn [167] and gemcitabine/carboplatin [168]. However, bortezomib in combination with erlotinib, which targeted EGFR mutations in NSCLC, did not show any survival benefit in patients with relapsed/refractory advanced NSCLC [169]. To date, bortezomib is not warranted for treating NSCLC patients in clinical practice; therefore further studies are needed to investigate the feasibility and validity in NSCLC patients.

TAK-243 (formerly known as MLN7243), as the primary mammalian E1 enzyme, is the first-in-class inhibitor of the UAE. TAK-243 treatment led to the depletion of cellular ubiquitin conjugates, resulting in disruption of signaling events in primary human xenograft [12]. Due to its specificity and potency, TAK-243 provides a new opportunity for UAE inhibition in cancer treatment. In addition, CC0651 is a small molecule inhibitor that selectively inhibits the E2 ubiquitin conjugating enzyme hCdc34 [170], but there is still a lack of preclinical or clinical information on CC0651 in lung cancer.

Likewise, DUB inhibitors targeting UPS have also become very attractive anticancer drugs and many of them have been investigated in preclinical studies. Pimozide and GW7647 are two potent and highly selective reversible inhibitors of the enzymatic activity of the USP1/UAF1 complex due to its involvement in translation synthesis and DNA damage response in NSCLC [22, 171, 172]. b-AP15 (also known as VLX1500) inhibited the activity of the deubiquitinases, ubiquitin C-terminal hydrolase 5 (UCHL5) and USP14, inducing tumor cells apoptosis and inhibiting tumor progression [173]. However, there still lacks information about drug efficacy and side effects to support the use of these inhibitors in clinical practice. Therefore, it is still too early to predict the therapeutic potential of DUBs in NSCLC and further ground-breaking developments might be obtained in the arenas of DUB biology and drug discovery in the future.

The article "The ubiquitin system: orchestrating cellular signals in non-small-cell lung cancer" was published in 2020. Journal: Cell Mol Biol Lett.

Despite these inhibitors showing promising prospects for clinical application, there are still a number of potential risks and problems to be solved. The ubiquitin system as an enormous biological regulator for thousands of genes plays a critical role in control of cellular signaling networks which affect a variety of phenotypes and biological process of tumor cells. Thus, in the development of new anti-cancer drugs in association with the ubiquitin system, the regulatory mechanisms of tumor related agents and the impacts on cell signaling still need to be described in-depth to effectively utilize the chemical inhibitors for therapy in cancer patients.

## Data Availability

Not applicable.

## Abbreviations

4E-BP1: 4E binding protein 1
APC/C: Anaphase-promoting complex/cyclosome
CHIP: Carboxy terminus of Hsc70 interacting protein
DAXX: Death domain-associated protein
DUBs: Deubiquitinating enzymes
EGF: Epidermal growth factor
EGFR: Epidermal growth factor receptor
GPCRs: G protein-coupled receptors
HECT: Homologous to E6-AP COOH terminus
IGF-1: Insulin-like growth factor-1
ILVs: Intraluminal vesicles
MJD: Machado-Joseph disease proteases
mTOR: Mammalian target of rapamycin
MVBs: Multivesicular bodies
NSCLC: Non-small-cell lung cancer
OTU: Ovarian tumor-like proteases
PI3K: Phosphoinositide-3-kinase
PKB: Protein kinase B
PKC: Protein kinase C
PTMs: Post-translational modifications
RBR: RING-between-RING
RCE1: Ras-converting enzyme 1
RING: Really Interesting New Gene
RTKs: Receptor tyrosine kinases
shh: Sonic hedgehog homolog
Smurf2: Smad ubiquitination regulatory factor 2
TNF: Tumor necrosis factor
TRAIL: TNF-related apoptosis-inducing ligand
TSC: Tuberous sclerosis complex
UAE: Ubiquitin activating enzyme
UAF1: USP1-associated factor 1
UCH: Ubiquitin carboxyl-terminal hydrolases
UCHL5: Ubiquitin C-terminal hydrolase 5
UPS: Ubiquitin-proteasome system
